# Deep parallel contextual analysis framework based emotion prediction in community wellness communications on social media

**DOI:** 10.1016/j.heliyon.2024.e31626

**Published:** 2024-05-21

**Authors:** Feng Liu, Kun Hou, Yang Dong

**Affiliations:** a School of Law, WeiFang University, Shandong, WeiFang, 261061, China; b Weifang Municipal Government Hospital, Department of Ultrasound, Shandong, WeiFang, 261041, China; c Weifang People's Hospital, Department of Radiology, Shandong, WeiFang, 261000, China

**Keywords:** Emotion prediction, Community wellness communications, Social media, Convolutional neural networks, Bidirectional long short-term memory network, Attention model, Text mining

## Abstract

Understanding public emotion on social media about community wellness is crucial for enhancing health awareness and guiding policy-making. In order to more fully mine the deep contextual semantical information of short texts and further enhance the effectiveness of emotion prediction in social media, we propose the Deep Parallel Contextual Analysis Framework (DPCAF) in the community wellness domain, specifically addressing the challenges of limited text length and available semantical features in social media text. Specifically, at the embedding layer, we first utilize two different word embedding techniques to generate high-quality vector representations, aiming to achieve more comprehensive semantical capture, stronger generalization ability, and more robust model performance. Subsequently, in the deep contextual layer, the obtained representations are fused with POS and locational representations, and processed through a deep parallel layer composed of Convolutional Neural Networks and Bidirectional Long Short-Term Memory Network. An attention model is then used to further extract semantical features of social media texts. Finally, these deep parallel contextual representations are post-integrated for emotion prediction. Experiments on a dataset collected from social media regarding community wellness demonstrate that compared to benchmark models, DPCAF achieves at least a 4.81 % increase in Precision, a 3.44 % increase in Recall, and a 10.81 % increase in F1-score. Relative to the most advanced models, DPCAF shows a minimum improvement of 2.65 % in Precision, 3.02 % in Recall, and 2.53 % in F1-score.

## 1 Introduction

In the digital era, social media has emerged as a crucial platform for disseminating community wellness information, significantly influencing public behaviors and attitudes towards health. The analysis of social media discourse in community wellness offers a key avenue for understanding and evaluating the impact of this information dissemination. By examining these social media posts, one can assess the reach of the information, public reactions, and the overall influence of these messages. This assists health organizations in refining their communication strategies, thereby enhancing the effectiveness of public health education.

Additionally, such analysis is vital for promptly identifying and rectifying erroneous or misleading information, ensuring the accuracy of health information provided to the public, and playing a critical role in responding to public health emergencies. In detail, it is not difficult to observe that the emotional elements carried in users' social media posts not only affect the breadth and depth of dissemination but also influence the emotions of other users. This can lead to a rapid accumulation of certain emotions in a short period, potentially triggering a burst in public opinion. Particularly in the case of destructive events concerning public safety, the asymmetry of information in public discourse often leads to social panic.

For instance, in 2020, due to the coronavirus disease 2019 (COVID-19) pandemic, many countries banned grain exports. Despite China's sufficient grain reserves at the time, rumors about a grain shortage still sparked a domestic frenzy of hoarding rice and flour. Therefore, it is essential to incorporate emotion prediction of social media discourse into the management of public emergencies. Identifying the emotional tone of social media discourse, understanding public attitudes and reactions to certain events, and using this understanding to effectively intervene and guide social media narratives are of great importance in fostering the positive development of public opinion.

Due to the length constraints and colloquial nature of social media texts, the available feature information is quite limited, making emotion analysis of social media far more challenging than that of standard texts. Therefore, a primary focus of current research is how to utilize deep learning models to fully extract more semantical information from social media texts. Traditional emotion prediction methods primarily include those based on emotion lexicons and machine learning techniques. The lexicon-based approach mainly involves matching against rules and emotion lexicons to analyze emotional tendencies. machine learning methods typically use annotated data to train classification models for predicting emotion categories.

In lexicon-based approaches, using the WordNet emotion lexicon, document [1] determined textual emotional tendencies by calculating the emotion scores of opinion words. Document [2] built a social media emotional lexicon on top of HowNet, incorporating social media linguistic features and introduced a sliding window to compute a subjectivity tendency coefficient for emotional classification of social media texts. Document [3] developed a emotional lexicon based on topic modeling, characterized by language independence, fine granularity, and unlimited capacity. Although simpler, lexicon-based methods require substantial effort in lexicon construction, and their quality and coverage directly affect emotion prediction accuracy.

In traditional machine learning-based methods, document [4] conducted emotion prediction comparative experiments using Naive Bayes, Maximum Entropy, and Support Vector Machines(SVMs). Document [5] incorporated Boosting techniques into Support Vector Machine classifiers and found improved performance. Document [6] combined classification rules, supervised learning, and machine learning to enhance emotion prediction results. Document [7] proposed a hierarchical multi-strategy social media emotion prediction method, including social media links and emoticons as feature information. Compared to lexicon-based methods, traditional machine learning approaches show improvement in effectiveness but require extensive manual annotation of training data.

In recent years, deep learning has increasingly become the mainstream method for emotion prediction. Compared to traditional machine learning models, this approach automatically extracts textual features during the training process, uncovering deeper semantic information through neural network models. Convolutional Neural Networks (ConvNets) are commonly used in emotion prediction. Document [8] used this model for short text emotion prediction, achieving an accuracy of 74.50 %. Zeng et al. proposed an improved ConvNet model, which performed well in aspect-level emotion prediction. Document [9] compared Vanilla Recurrent Neural Network (RNN), Long Short-Term Memory (LSTM), and Gate Recurrent Unit (GRU) in emotion prediction, finding that GRU outperformed the other two models, with an 8.62 % increase in accuracy over RNN.

To better learn phrase-level dependencies, document [10] used RNN and AdaRNN to build phrase-level RNN for emotion prediction. Document [11] proposed a C-LSTM model based on ConvNet and LSTM, where the text features extracted by ConvNet are processed by LSTM replacing the ConvNet pooling layer, showing superior performance over ConvNet and LSTM. Document [12] proposed a neural network based on an emotion information collector and extractor, utilizing the Bidirectional Long Short-Term Memory (Bi-LSTM) model to generate an information matrix as the input for the extractor. This approach achieved an accuracy of 84.36 % on the Sina microblog social media dataset.

In summary, emotion prediction has gradually shifted from traditional methods based on emotion lexicons and machine learning to emerging approaches centered around deep learning. However, existing Chinese social media emotion prediction often relies on a single feature representation, failing to fully exploit the advantages of multi-feature and multi-channel models in extracting multi-layered emotional features and overlooking the subtle emotion information present in short texts, such as word classes and location. Addressing these issues and the limitations of text length and available feature information in social media, we propose a deep parallel contextual analysis framework based emotion prediction in community wellness communications on social media.

This model, by introducing the multi-feature integration-based deep contextual layer and multi-channel-based deep parallel strategy building upon ConvNet and Bi-LSTM frameworks with an integrated attention model, more effectively mines deep semantical information in social media short texts, thereby further enhancing the effectiveness of emotion prediction on social media.

Our study aims to establish a more robust understanding of public emotion dynamics in community wellness discussions on social media platforms, thereby fostering health awareness and informing policy-making initiatives. By introducing the Deep Parallel Contextual Analysis Framework (DPCAF), we seek to address the pressing challenge of efficiently extracting deep contextual semantic insights from brief social media posts to enhance emotion prediction accuracy. Through the integration of novel methodologies, our framework transcends the constraints posed by text length and available semantic features, offering a comprehensive solution for analyzing sentiment in community wellness discourse.

Furthermore, our research contributes to the scientific community by presenting a methodological advancement in the domain of social media sentiment analysis. The innovative combination of multi-feature integration-based deep contextual layers and multi-channel-based deep parallel strategies, underpinned by ConvNet and Bi-LSTM frameworks with an integrated attention mechanism, represents a significant step forward in sentiment analysis methodology.

## 2 Related works

This section will introduce related emotion prediction methods in social media, starting with traditional emotion prediction approaches, which include lexicon-based, machine learning-based, and deep learning-based methods. However, these methods have limited contextual understanding, especially lexicon-based and traditional machine learning approaches. As a Transformer-based model, BERT (Bidirectional Encoder Representations from Transformers) employs bidirectional context to comprehend text, meaning it considers all words before and after each word in the text for a more comprehensive understanding of language. Hence, we also introduce emotion prediction methods based on the BERT model.

### 2.1 Traditional emotion prediction approaches

#### 2.1.1 Lexicon-based emotion prediction methods

Lexicon-based emotion prediction simply involves matching pre-processed words with those in a emotional lexicon and calculating a emotion score based on the degree of matching to determine emotion polarity. This method is computationally straightforward and does not require additional resources. Representative studies on lexicon-based emotion prediction, as discussed in the document [13], focus on the construction of emotion lexicons. These lexicons comprise a collection of nouns, verbs, adjectives, and adverbs with fixed emotional tendencies, such as positive words like *joy, happily, hero*, and negative ones like *sad, sadly, traitor*. The widely used Chinese emotion lexicons include HowNet's [14], National Taiwan University's NTUSD [15], and Dalian University of Technology's ontology library [16].

The construction of emotion lexicons is a labor-intensive and complex task. Traditional methods for building these lexicons are mostly based on semantical similarity, where the core idea is to measure the distance between candidate words and positive/negative emotion labels, generally using Point-wise Mutual Information (PMI) as the measurement method. Document [17] based their emotion lexicon on topic models. With the rapid development of artificial intelligence in recent years, many have started using machine learning-based methods [18] and deep neural network-based methods [19] to construct emotion lexicons.

To enhance the expression of emotions, users often utilize emotionally strong symbols in their social media posts, such as emojis, popular internet slang, adverbs of emotion, or degree. Therefore, it is crucial to consider the role of these emotional symbols when analyzing the emotion of social media content. Document [20] elaborates on the importance of emotional symbols and how to analyze the emotion of social media content based on these symbols.

While lexicon-based emotion prediction methods are simple to operate, their accuracy in emotional classification is generally lower compared to machine learning-based and deep learning-based methods. This is mainly because: (1) The construction of emotion lexicons is challenging, and the lexicons built are generally applicable within a specific domain, which makes lexicon-based methods less versatile and robust. (2) Chinese texts often exhibit phenomena like polysemy and irony, where the same word may have different emotional tendencies in different contexts. Additionally, the timeliness of social media corpus is strong, and new internet slang words emerge daily. If the emotion lexicon is not updated promptly, it might incorrectly judge the emotional tendencies of these words, leading to significant deviations in analysis results.

#### 2.1.2 Machine learning-based emotion prediction methods

Machine learning-based emotion prediction methods involve feature selection from a large corpus, primarily through manual screening, followed by representing the entire text with selected features and classifying the text using machine learning algorithms. These emotion prediction methods can be divided into supervised and unsupervised approaches.

(1) Supervised machine learning methods

For emotion prediction using supervised machine learning, extensive manual labeling of social media data is required, where each post's emotional tendency is annotated. This labeled data is then used as a training set for text classification. Common classification methods include Naive Bayes (NB), SVM, Maximum Entropy (ME), K-Nearest Neighbors (KNN), and Conditional Random Fields (CRF). Document [21] used movie reviews as base data and applied NB, ME, and SVM classifiers for binary classification of review data. Document [22] also treated emotion prediction as a binary classification problem, employing NB, SVM, and Recchio methods for emotion classification, along with Chi-square (Chi) and Information Gain (IG) for feature selection.

Document [23] compared emotion prediction methods such as NB, SVM, and N-Gram on a travel blog comment dataset, finding that SVM and N-Gram outperformed NB. Document [24] compared SVM and CRF using a web blog corpus, demonstrating that CRF's classification results were superior to SVM's. Document [25] described the Multimodal Joint Sentiment Topic Model (MJST), a novel approach for weakly supervised sentiment analysis on microblogging platforms. This model uniquely integrated Latent Dirichlet allocation (LDA) [26] to analyze sentiments and topics by incorporating multimodal features like emoticons and aspects of microbloggers' personalities.

(2) Unsupervised machine learning methods

Although supervised machine learning methods offer higher accuracy, they heavily rely on manually labeled data, which is not only labor-intensive but also prone to inconsistencies. Unsupervised machine learning methods, in contrast, do not require manual labeling, though their accuracy is generally lower. For emotion prediction using unsupervised approaches, it is common to select benchmark emotion words and then conduct topic segmentation. Popular methods include Probabilistic Latent Semantic Analysis (PLSA) [27] and LDA. PLSA and LDA are typically used for document-level long texts and are not well-suited for short texts like posts. To address this, document [28] proposed the Biterm Topic Model (BTM) specifically for short text topic modeling, explicitly establishing a pattern of word co-occurrence.

The research on Chinese microblog emotion prediction using machine learning started later compared to English and is relatively behind in terms of research resources and methodologies. This is primarily due to several reasons: Chinese texts require word segmentation before emotion prediction; Chinese language is characterized by a high occurrence of polysemy, positive and negative connotations; and the context in Chinese texts is more interrelated. Targeting Chinese texts, document [29] used CRF to capture the contextual constraints of sentence emotions, introducing redundant features to capture the overlapping tags between emotional categories. Document [30] studied three classification methods in Chinese, i.e., NB, EM, and SVM, and combined them using Stacking for classification in different domains.

#### 2.1.3 Deep learning-based emotion prediction methods

Compared to machine learning-based methods, deep learning-based approaches do not require manual feature extraction. They can automatically extract primary features and combine them into higher-level features for automatic emotion classification. Among various neural network models suitable for emotion prediction, the primary ones are ConvNet and RNN.

ConvNet is a type of neural network that computes local features using convolutional kernels. ConvNets have the capability to hierarchically extract features and can perform multi-level deep combinations, often used in image recognition. Document [31] introduced TextCNN for text classification, where text data is mapped into word vectors through word embeddings and then formed into a matrix as the input for the ConvNet. This model's ConvNet architecture is relatively simple, comprising only one convolutional layer and one pooling layer, yet it achieved the best accuracy rates at the time on multiple datasets. Targeting social texts, document [32] trained word vectors at the word level and then fed these trained vectors into ConvNet for sentence feature extraction and emotion judgment, demonstrating that ConvNet can extract sentence features from short texts and is suitable for social emotional classification.

RNN consist of many sequentially computed neural network units, with each unit's input containing the output of the previous unit. This endows RNNs with memory, making them suitable for processing sequential data. Text data, such as *The cat eats the mouse* versus *The mouse eats the cat*, though containing the same words, have entirely different meanings due to the sequence of words.

Fig. 1 illustrates the process of emotion prediction based on RNN, where each neural unit in the RNN sequentially reads text information. Each *ℎ*_*i*_ is a hidden output unit containing information from *ℎ*_*i-*1_, meaning the last hidden output unit *ℎ*_*N*_ contains semantic information from all previous text. Finally, the classifier determines the emotion based on the information in *ℎ*_*N*_.

**Fig. 1:** Emotion prediction process based on RNN.

### 2.2 BERT-based emotion prediction methods

#### 2.2.1 Introducing attention model in emotion prediction

Deep learning-based emotion prediction methods typically encode text as a whole, failing to fully consider the effects of emotional symbols. In contrast, lexicon-based emotion prediction methods overly rely on emotional factors and do not adequately consider the semantical relationships within the entire text. Additionally, deep learning-based methods usually analyze single posts, neglecting the global text structure and emotional factors. To address these issues, many researchers have introduced attention models into emotion prediction. This subsection summarizes the use of attention models in emotion prediction in recent years, as shown in Table 1.

**Table 1:** Emotion prediction methods based attention and deep learning.

Documents	Attention model	Network model
[33]	Bi-self attention model	LSTM
[34]	Multi-head attention model	Bi-LSTM
[35]	Bi-level attention (word level, sequence level)	Theme model
[36]	Feature enhanced attention	ConvNet, Bi-LSTM
[37]	Dual attention	Custom deep learning model
[38]	Global attention, local attention	Bi-LSTM
[39]	Word level attention	GRU
[40]	Hierarchical attention	Bi-GRU
[41]	Topic-level attention	Emotion-enhanced LSTM
[42]	Original attention	LSTM

#### 2.2.2 Transformer model

The Transformer model, proposed by Ref. [43], is an Encoder-Decoder model implemented with Self-Attention. Typically, the core structure of Encoder-Decoder models is based on RNN, but RNN has issues like inability to parallelize computations and susceptibility to gradient vanishing or exploding. Therefore, the Transformer model uses Self-attention in place of traditional RNNs.

As shown in Fig. 2, the input to the Encoder is the word vector representation of a sentence, added with position encoding information of the sentence. It then passes through a Self-Attention layer, which helps the Encoder to see the information of words before and after each word during encoding. The output of the Self-Attention layer goes into an Add & Norm layer, where Add means adding the input and output of the Self-Attention layer, and Norm refers to normalizing the added output. The normalized result is then fed into a fully connected feed-forward neural network, followed by another Add & Norm operation. The most crucial part of the BERT model is based on the aforementioned type of Encoder.

**Fig. 2:** Encoder of transformer.

#### 2.2.3 BERT model

BERT, introduced by Ref. [44], is a language model based on the bidirectional Transformer model, as shown in Fig. 3, where ***E***_1_, ***E***_2_, …, ***E***_*N*_ represent inputs, and ***T***_1_, ***T***_2_, …, ***T***_*N*_ represent outputs.

**Fig. 3:** Bert.

The input to the BERT model is the sum of three vectors: word vectors, segment vectors, and location vectors. The word vector represents the encoding of the current word, the segment vector encodes the location of the current word in the sentence, and the location vector encodes the location of the current word, with each sentence using CLS and SEP as markers for the beginning and end.

To enhance the model's semantical representation capabilities, BERT innovatively proposes two pre-training tasks during its training: MLM (Masked LM) and NSP (Next Sentence Prediction). The MLM task involves randomly masking one or several words in a sentence and using the remaining words to predict them, typically masking 15 % of the words. The NSP task involves given two sentences from an article, determining whether the second sentence directly follows the first in the article. BERT has achieved good results in many NLP tasks, such as emotion classification and question-answering systems.

#### 2.2.4 Emotion prediction methods based on BERT

Using the BERT model for social emotion prediction is a downstream task of BERT, generally involving generating text vector representations with the pretrained BERT model, followed by emotion classification using relevant classification algorithms. Unlike word2vec, BERT generates word vectors dynamically, considering more comprehensively the information between semantics [45]. Table 2 summarizes recent methods using the BERT model for emotion prediction.

**Table 2:** Emotion prediction methods based BERT.

Documents	Details
[46]	Using the BERT model as the word embedding layer, then combining it with Linear, GRU, SAN, TFM, and CRF methods for emotion analysis experiments on two datasets from SemEval.
[47]	Proposing an improved BERT model - the RoBERT model.
[48]	Based on the RoBERT model, conducting emotion analysis on the 2019 CCF BDCI and 2019 CCKS datasets, identifying negative factors.
[49]	Using four methods for emotion analysis on a movie review dataset: lexicon-based, machine learning-based, deep learning-based, and BERT-based, with experiments showing the BERT-based method was most effective.
[50]	Proposing a BERT-based target-oriented multimodal emotion analysis model, TomBERT, and performing emotion analysis using the TomBERT model on a Twitter dataset.
[51]	Building a emotion classifier based on a pre-trained BERT model, performing aspect-oriented emotion analysis at both sentence and document levels.
[52]	Proposing a combination of BERT with Bi-LSTM and Bi-GRU to enhance accuracy and investigate the effects of hybridizing layers in BERT models (DistilBERT, RoBERTa) for text sentiment classification, both with and without emojis.
[53]	Introducing a single-stream transformer model, All-modalities-in-One BERT (AOBERT), pre-trained simultaneously on Multimodal Masked Language Modeling (MMLM) and Alignment Prediction (AP) to determine dependencies and relationships between modalities.
[54]	Proposing the BERT-GAN model with review aspect fusion to improve the fine-tuning performance of the BERT model. This approach incorporates semi-supervised adversarial learning, fusing service aspects from consumer reviews with word sequences before model input, enhancing aspect representation and positional context in sentences.
[55]	Proposing a hierarchical multi-head self-attention and gate channel BERT for optimized feature extraction and information filtering. This model consists of three modules: a hierarchical multi-head self-attention module for feature extraction, a gate channel module replacing BERT's original Feed Forward layer, and a tensor fusion model based on a self-attention mechanism for integrating different modal features.

## 3 Materials and methods

### 3.1 Foundation construction

#### 3.1.1 Word vector representation

Word vector representation involves converting text into a vector form. Word2Vec is a commonly used word vector model in emotion prediction, comprising CBOW (Continuous Bag-Of-Words) and Skip-Gram models. CBOW predicts the center word given the context words but ignores the impact of word order on semantics. In contrast, Skip-Gram, with the center word as input, predicts the context words, considering text order more thoroughly. FastText, building on Word2Vec, introduces character-level N-grams as additional feature inputs and employs hierarchical Softmax, significantly reducing model training time. GloVe learns word vectors based on statistical co-occurrence matrices, capturing global information, and is another commonly used word vector model.

#### 3.1.2 ConvNet

ConvNet, initially applied in image recognition tasks, is now widely used in emotion prediction research, showing significant advantages in hierarchical semantic information acquisition. ConvNet consists of an input layer, convolutional layers, pooling layers, and fully connected layers. The model first represents text sequences as vector matrices at the input layer; then, it employs convolutional kernels in the convolutional layer to extract features through one-dimensional convolution; next, it uses mean pooling or max pooling in the pooling layer for feature selection and filtering, outputting fixed-dimension matrices; finally, the fully connected layer concatenates the features after pooling.

#### 3.1.3 LSTM

LSTM is an improvement based on RNN. When dealing with long text sequences, RNN, due to gradient dispersion, captures only recent sequence information, losing a lot of early sequence information. LSTM resolves RNN's issues of gradient dispersion, explosion, and short-term memory by adding cell states and gate mechanisms.

LSTM comprises forget gates, input gates, and output gates. The forget gate decides whether to retain information through the Sigmoid function; the input gate filters incoming information, ignoring features with a zero output dimension, and updates the current cell state by combining temporary and previous cell states; the output gate selectively retains and ignores current moment information, calculating the output result through the tanh function, serving as input for the next moment.

#### 3.1.4 Bi-LSTM

Bi-LSTM is a variant of LSTM. It concatenates forward-propagating LSTM with backward-propagating LSTM, obtaining semantic features from both directions, effectively addressing context dependency issues.

#### 3.1.5 Attention model

The attention model, a method for extracting important data features, was initially applied in image processing tasks. Document [51] first proposed applying the attention model in natural language processing tasks to alleviate RNN's long-distance dependency issues. In emotion prediction, the attention model can address problems of establishing dependencies between source and target sequences due to excessive distance. Since the importance of words in a text varies, leading to different feature weights, introducing the attention model allows for better learning of word dependencies, enhancing focus on important words.

### 3.2 Model construction

#### 3.2.1 General framework

Our overall framework is depicted in Fig. 4. Initially, we obtain social data through web scraping, followed by preprocessing and part-of-speech (POS) tagging. Subsequently, Word2Vec and FastText are employed to generate word vectors from social text, which are then concatenated with POS feature vectors and location feature vectors. This process aims to fully mine the subtle emotional information contained in the emotional words and their positional relationships within the short social texts.

**Fig. 4:** Proposed DPCAF model.

Subsequently, these multi-feature integrated vectors, processed through the deep contextual layer, are input into the deep parallel multi-channel layer constructed using ConvNet and Bi-LSTM, followed by the introduction of an attention model [56]. This model effectively utilizes both global and local deep semantical features of social texts, thereby enhancing the emotion prediction performance.

#### 3.2.2 Model overview

In this paper, we propose a DPCAF model. This model has a 5-layer structure:

(1) Feature embedding layer (include feature extraction and deep contextual layer): Word2Vec and FastText are used to generate word vectors, which are then fused with POS feature vectors generated from POS information and position feature vectors generated from position information. This results in multi-feature integrated vectors, i.e., contextual feature vector of Word2Vec(CFVW) and contextual feature vector of FastText(CFVF).
(2) Deep parallel layer: CFVW and CFVF are used as inputs to construct four channels, employing ConvNet and Bi-LSTM to extract local and global semantical features.
(3) Attention model layer: An attention model is introduced after the multi-channel hybrid neural network model to fully consider the important semantical features in social texts.
(4) Integration layer: The local and global features extracted through the attention model layer are concatenated and integrated.
(5) Output Layer: The Softmax function is used to perform emotion prediction on the output features of the integration layer.

#### 3.2.3 Feature embedding layer

(1) POS Feature Vector

Due to the limited length of social posts, which often contain short texts and colloquial expressions, the useable feature information is very limited. To more fully mine the lexical feature information in social texts, we utilize the HowNet emotion lexicon and employ Jieba for part-of-speech tagging of 6 types of emotional words, as shown in Table 3. Specific emotional words appearing in social texts are transformed into *m*-dimensional continuous POS feature vectors to fully extract subtle emotional information from social texts. In the representation of POS feature vectors, the *i*-th word POS feature vector, *e*_*i*_ ∈ **R**^*m*^, is defined.

(2) Locational feature vector

**Table 3:** PART–OF–SPEECH labelling standards

Emotion word names	Part-of-speech labelling
Positive comment words	PC
Positive emotive words	PE
Negative comment words	NC
Negative emotive words	NE
Degree words	DW
Negation words	NW

In social texts, there is an interaction between emotional words, degree words, and negation words. The same word may express different degrees of emotion depending on its location, and the locational value varies accordingly. Locational value, a numerical representation of the relationship between words, is used to generate locational feature to better represent the importance of words in a sentence. The calculation of locational value is shown in equation (1):

(1) $$Location_{i}=\left\{ \begin{array}{c} \text{maxlen}-\text{len}\left(\text{words}\right)+i,e_{i}=0\\ \text{maxlen}+i,e_{i}\neq 0 \end{array}\right.$$

where Location_*i*_ denotes the locational value of the *i*-th word in the text sequence; *e*_*i*_ ≠ 0 indicates that the word contains part-of-speech features; maxlen is the maximum step length of the input text sequence; len(words) is the length of the text sequence. Similar to the method for generating POS feature vector, each locational value in this paper is transformed into an *r*-dimensional continuous location feature vector. In the representation of the location feature vector, the *i-*th word location feature vector is defined as *p*_*i*_ ∈ **R**^*m*^.

(3) Multi-feature integration vector

To more fully consider the semantical connections between features, the word vectors generated by Word2Vec and FastText are fused with POS feature vector and location feature vector to create multi-feature fusion vectors CFVW and CFVF. The integration calculation is shown in equations (2), (3), (4), (5):

(2) $$x_{wep_{i}}=\mathrm{Int}\left(v_{wi},e_{i},p_{i}\right)\in R^{d+m+r}$$

(3) $$X_{wep}=\left[x_{wep_{1}},x_{wep_{2}},...,x_{wep_{n}}\right]$$

(4) $$x_{fep_{i}}=\mathrm{Int}\left(v_{fi},e_{i},p_{i}\right)\in R^{d+m+r}$$

(5) $$X_{fep}=\left[x_{fep_{1}},x_{fep_{2}},...,x_{fep_{n}}\right]$$

where *Int* denotes the integration operation and *n* is the length of the text sequence. These equations and processes describe the comprehensive approach of integrating various feature vectors to enrich the semantic analysis capabilities. The specific process is illustrated in Fig. 5. Firstly, the *i*-th word is transformed into a dimension *d* word vector matrix *v*_*wi*_ and *v*_*fi*_ by Word2Vec and FastText, respectively. Then, it is fused with the POS feature vector *e*_*i*_ and location feature vector *p*_*i*_, generating a dimension *d + m + r* multi-feature integration vector matrix *x*_*wepi*_ and *x*_*fepi*_. Finally, the word-level features are concatenated into sentence-level features as input for the next layer.

**Fig. 5:** Integrating contextual feature vector.

#### 3.2.4 Deep parallel layer

The deep parallel layer further extracts features from the fused vectors. In this layer, CFVW is fed into ConvNet and Bi-LSTM, as is CFVF, forming four channels to extract local and global features from the previous layer of the model.

The neural network structure based on CFVW is shown in Fig. 6, with the CFVF-based structure being similar. On one hand, convolution operations are performed using convolutional kernels of different sizes to generate three types of feature maps, followed by a max-pooling strategy to obtain a comprehensive set of local features. On the other hand, Bi-LSTM is used to extract and concatenate the emotional features from both forward and reverse directions, thereby acquiring the global context features. The computations are as shown in equations (6), (7), (8), (9), (10), (11), (12), (13), (14), (15).

(6) $$\begin{array}{c} X_{1:n}=\left[x_{1},x_{2},...,x_{n}\right]\\ s.t.x_{i}\in R^{d+m+r} \end{array}$$

(7) $$C_{h_{s}}=\text{Relu}\left(W_{s}X_{i\to i+h_{s}-1}+b_{s}\right)$$

(8) $${\dot{C}}_{h_{s}}=\max\left(C_{h_{s}}\right)$$

(9) $$v_{h_{s}}=Con\left({\dot{C}}_{h_{s1}},{\dot{C}}_{h_{s2}},...,{\dot{C}}_{h_{sm}}\right)$$

(10) $$x_{i}v_{i}=\left[v_{h_{1}},v_{h_{2}},v_{h_{3}}\right]$$

(11) $$H_{c}=\left[v_{1},v_{2},...,v_{n}\right]$$

(12) $$h_{F}=F-LSTM\left(x_{i}\right)$$

(13) $$h_{B}=B-LSTM\left(x_{i}\right)$$

(14) $$h_{i}=\left[h_{F},h_{B}\right]$$

(15) $$H_{b}=\left[h_{1},h_{2},...,h_{n}\right]$$

**Fig. 6:** Integrated neural network model.

In which, *x*_*i*_ is the vector of the *i*-th word, *W*_*s*_ is the convolutional kernel, *h*_*s*_ is the size of the convolutional kernel window (1 ≤ s ≤ 3), *b*_*s*_ is the bias term, *m* is the number of convolutional kernels, Relu() is the activation function; *H*_*c*_ is the feature of the ConvNet channel. In adition, F-LSTM() refers to forward-propagating LSTM; B-LSTM() refers to backward-propagating LSTM, *h*_*s*_ is the concatenation result of *ℎ*_*F*_ and *ℎ*_*B*_, *H*_*b*_ is the feature of the Bi-LSTM channel.

#### 3.2.5 Attention layer

Given the attention model's favorable performance in machine translation, entity recognition, and sequence tagging tasks, we introduce it after the deep parallel layer in our framework. The model weights the vectors to extract important features. Specifically, the hidden layer vector *h*_*i*_ is first fully connected using the non-linear activation function tanh to obtain *u*_*i*_. next, softmax function normalizes it to learn each word's attention weight *α*_*i*_*.* Finally, the weight *α*_*i*_ is applied to the corresponding hidden layer vector *h*_*i*_ in a weighted sum to produce the attention output *H*_*a*_, as shown in equations (16), (17), (18).

(16) $$u_{i}=\tanh\left(W_{w}h_{i}+b_{w}\right)$$

(17) $$\alpha_{i}=\text{softmax}\left(u_{i}\right)$$

(18) $$H_{a}=\sum_{i}\alpha_{i}h_{i}$$

#### 3.2.6 Integration layer

The proposed DPCAF integration layer combines features output from the deep parallel layer to create a contextual vector, which utilizes the multi-layer semantical information of social texts. Specifically, local features are obtained through iterative calculations by ConvNet, global features are obtained using Bi-LSTM combined with sequence information. Finally, the attention model is introduced for a secondary extraction to retain important features.

During model training, binary cross-entropy is used as the loss function, as shown in equation (19):

(19) $$Loss=-\sum_{i=1}^{D}\sum_{k=1}^{C}y_{i}^{k}\;\log\left(p_{i}^{k}\right)$$

Here, *i* is the index of the social text sequence, *k* is the index of the emotion category, *D* is the size of the training dataset, *C* is the number of categories, *p* is the predicted category probability, and *y* is the actual category.

#### 3.2.7 Output layer

Based on the feature vectors extracted from the integration layer, the output layer employs the Dropout mechanism to randomly select neurons to drop, combining the result with softmax to perform emotional classification. The classification prediction is calculated as shown in equation (20).

(20) Y=argmax(softmax(WH+b))

In which, *H* is the feature vector extracted from the integration layer, *Y* is the predicted category.

## 4 Experiments and results

### 4.1 Collection and processing of data set

Sina microblog is a microblogging platform that offers users the convenience to post or access information online. Through WEB, WAP, and other client applications, general users can publish messages on Sina microblog at any moment, usually not exceeding 140 characters, or by means of images and short videos. Owing to its user-friendly and rapid nature, Sina microblog has garnered a vast user base. Official statistics indicate that as of March 2020, Sina microblog's monthly active users have reached 550 million, with daily active users at 241 million, marking an increase of 85 million and 38 million, respectively, compared to the same period of the previous year. Thus, it is evident that Sina microblog has become one of the primary channels for the public to post comments online and express their viewpoints and demands.

Taking the public health emergency of the COVID-19 outbreak as an example, we utilized a combination of Beautiful Soup and Requests, a scraping toolset that uses Python's Requests library for HTTP requests and Beautiful Soup for page parsing. Specifically, with keywords like COVID-19 and novel coronavirus, we scraped Sina microblog posts from February 1, 2020, to December 31, 2020, yielding 165,882 data entries. To ensure the reliability of data quality, stringent pre-processing was conducted on the experimental data, removing duplicates and low-quality posts, and minimizing the impact of class imbalance, ultimately obtaining a balanced dataset of 157,174 posts, with 78,587 entries in both positive and negative categories. Semi-automated annotation processes were employed, along with multiple rounds of labeling to guarantee the reliability and validity of the data.

Specifically, iFlytek's API was first used to label the emotional polarity of the preprocessed data; then, manual verification of the labeling results was conducted to determine the final annotation values. This data was used for both model training and vector generation, with examples of the annotations provided in Table 4.

**Table 4:** Example presentation of the dataset.

Emotional polarity	Texts
Positive class/1	["They have been very successful in fighting the epidemic” #New York Times Reporter Praises China's Epidemic Battle#] “China has been very successful in fighting the epidemic!” “Don't think the cabin hospital dances are ridiculous; they are a clever healing method” “Isolation is the trick for China to block the epidemic transmission,” says Donald McNeil, a senior health and science reporter for The New York Times. Recently, he publicly praised China's “epidemic battle,” corrected the distortions and misunderstandings of Western media, and believed it formed a stark contrast with the responses of Italy and the United States. This video has already been watched and shared by millions of people worldwide. (In Chinese)
Negative class/0	[#The pathogen of Wuhan pneumonia epidemic is not the SARS virus#] In recent days, the claim that the Wuhan pneumonia epidemic is caused by a new SARS virus has been circulating online. On January 18, the Chinese Center for Disease Control and Prevention's official account published a science popularization article “Don't Believe These 5 Major Rumors About the Viral Pneumonia in Wuhan!” The article mentioned that the pathogen causing the Wuhan viral pneumonia epidemic is not the SARS virus. Current investigations show that this virus's ability to transmit between people and its pathogenicity are both weaker than SARS. #Wuhan reports 4 new cases of novel coronavirus pneumonia#. (In Chinese)

### 4.2 Evaluation metrics

In our emotion prediction experiment, we use Precision, Recall, and F1-Score as the model evaluation metrics, as shown in equations (21), (22), (23):

(21) $$\text{Precision}=\frac{TP}{TP+FP}$$

(22) $$\text{Recall}=\frac{TP}{TP+FN}$$

(23) $$F1-\text{Score}=2*\frac{\text{Precision}*\text{Recall}}{\text{Precision}+\text{Recall}}$$

In which, *TP* represents the number of positive class samples correctly predicted as positive, *FP* represents the number of negative class samples incorrectly predicted as positive, *FN* represents the number of positive class samples incorrectly predicted as negative.

### 4.3 Experiment settings

The experimental environment is as follows: Intel® Core™ i5-9400 F CPU, GeForce RTX 2060 GPU, with a core frequency of 1365 MHz, memory frequency of 14,000 MHz, 6 GB of RAM, running on Windows 11 OS. The development environment is Anaconda + pytorch1.13.1 + CUDA11.7 + cuDNN8.9 +Python 3.9. In addition, the specific parameter settings and descriptions of the model are shown in Table 5.

**Table 5:** Parameter setting of the model.

Parameter names	Values
Maximum length of text sequences	200
Dimension of word vectors	100
Dimension of part-of-speech feature vectors	30
Dimension of location feature vectors	20
Batch size	256
Convolutional kernel window size	3,4,5
Number of convolutional kernels	100
Hidden layer size of Bi-LSTM	256
Epochs	10
Learning rate	0.01
Dropout	0.5
Optimizer	Adam
Training/testing/validation set splitting protocol	8:1:1

### 4.4 Contrast experiments

In this section, we explore the comparative effectiveness of emotion prediction across different models. Specifically, we conduct a comparative analysis of five benchmark models: SVM [30], ConvNet [8], RNN [10], LSTM [11], and Bi-LSTM [12], as well as three advanced models, namely ConvNet&Bi-LSTM [36], Hybrid attention network [38], and Self-adapting BERT [50] (their introductions can be found in the related work section), in comparison with the proposed model. The experimental results are presented in Table 6.

Firstly, it is evident that the proposed method, along with other advanced methods, significantly outperforms the naive benchmark approaches. For instance, ConvNet&Bi-LSTM shows at least a 1.33 % increase in Precision, a 7.73 % increase in Recall, and a 2.62 % increase in F1-Score over Bi-LSTM.

Secondly, in the comparison of our method with these advanced methods:

(1) Compared to ConvNet&Bi-LSTM, our method shows a 3.48 % improvement in Precision, a 0.56 % improvement in Recall, and an 8.19 % improvement in F1-Score. This is attributed to the proposed method's integration of Word2Vec and FastText generated word vectors with deep contextual fusion of part-of-speech and locational features, coupled with the parallel application of ConvNet and Bi-LSTM. This not only enhances the capture of local and global features but also deepens the semantical understanding of the text. The combined feature extraction and enhanced semantical representation are the primary reasons for its superiority in Precision and F1-Score over ConvNet&Bi-LSTM.
(2) In comparison to the Hybrid attention network, our method shows a 2.86 % higher Precision, a 4.56 % higher Recall, and a 3.68 % higher F1-Score. By integrating different types of word vectors and feature vectors, and employing a parallel structure with attention models, our method effectively improves the ability to capture the emotion tendencies in social media text. This approach is more effective than the singular use of global or local attention models, especially in handling complex texts with noise targets.
(3) Relative to Self-adapting BERT, our method achieves a 2.65 % improvement in Precision, a 3.02 % improvement in Recall, and a 2.53 % improvement in F1-Score. While the BERT model has made significant advances in emotion prediction, it has limitations in interpretability and integration of specific emotion knowledge. Our approach combines deep learning with granular analysis of part-of-speech and positional features, enhancing the model's sensitivity to emotion tendencies, particularly effective when the data size is relatively small.

### 4.5 Ablation experiments

#### 4.5.1 Impact of deep contextual layer

This section explores the impact of deep contextual integration on emotion prediction. Firstly, we compare the experimental effects of three models: Word2Vec, FastText, and GloVe. Then, based on the two superior models from these results, we generate word vectors and integrate part-of-speech and locational features to create deep contextual integration vectors, i.e., CFVW and CFVF. Finally, we analyze the impact of deep contextual integration on different models using Bi-LSTM and ConvNet, as shown in Table 7.

Based on Table 6, Table 7, different vector representations significantly impact experimental results. In terms of F1-score, ConvNet&Word2Vec and ConvNet& FastText outperform ConvNet&GloVe by 0.17 % and 0.22 %, respectively, and ConvNet by 1.41 % and 1.46 %, respectively. Bi-LSTM&Word2Vec and Bi-LSTM& FastText exceed Bi-LSTM&GloVe by 0.18 and 0.41 %, respectively, and Bi-LSTM by 3.51 and 3.73 %, respectively. This suggests that word vectors generated by Word2Vec and FastText achieve better results than GloVe and random vectors, indicating that the initial values of feature vectors influence experimental outcomes. Therefore, Word2Vec and FastText are selected for subsequent deep contextual integration operations in this paper.

**Table 6:** Comparative experimental results.

Methods	Precision(%)	Recall (%)	F1-socre (%)
SVM	74.12	67.43	71.34
ConvNet	78.27	76.88	76.59
RNN	78.65	79.71	75.45
LSTM	78.98	72.6	73.82
Bi-LSTM	80.62	80.33	75.34
ConvNet&Bi-LSTM	81.95	83.21	77.96
Hybrid attention network	82.57	79.21	82.47
Self-adapting BERT	82.78	80.75	83.62
**DPCAF**	**85.43**	**83.77**	**86.15**

**Table 7:** Results of ablation experiments on deep contextual integration.

Methods	Precision(%)	Recall (%)	F1-socre (%)
ConvNet & GloVe	79.28	77.4	77.83
ConvNet & Word2Vec	79.92	77.3	78
ConvNet & CFVW	79.62	78.12	78.43
ConvNet & FastText	79.33	77.28	78.05
ConvNet & CFVF	80.06	78.40	78.87
Bi-LSTM & GloVe	79.95	78.15	78.66
Bi-LSTM & Word2Vec	79.99	78.35	78.85
Bi-LSTM & CFVW	80.1	79.78	79.84
Bi-LSTM & FastText	79.76	78.26	79.07
**Bi-LSTM & CFVF**	**80.19**	**80.91**	**79.35**

It is also observed that Bi-LSTM outperforms ConvNet with the same word vector input. In terms of F1-score, Bi-LSTM&Word2Vec improves upon ConvNet&Word2Vec by 0.85 %, and Bi-LSTM&FastText improves upon ConvNet&FastText by 1.02 %. This is attributed to the complex expressions and colloquial language in microblog texts. ConvNet fails to fully learn semantic information, while Bi-LSTM accounts for the impact of word order on semantics, resulting in better performance.

Further analysis reveals that models with deep contextual integration vectors outperform those with single word vectors. Specifically, in terms of F1-score, ConvNet&CFVW improves upon ConvNet&Word2Vec by 0.43 %, ConvNet&CFVF improves upon ConvNet&FastText by 0.82 %, Bi-LSTM&CFVW improves upon Bi-LSTM&Word2Vec by 0.99 percentage points; and Bi-LSTM&CFVF improves upon Bi-LSTM&FastText by 0.32 %.

These results indicate that compared to single word vectors and random vectors, proposed deep contextual integration vectors can effectively learn semantic connections between features and utilize part-of-speech and locational information, thereby enhancing model performance.

#### 4.5.2 Impact of attention model

In this section, we explore the impact of attention model on emotion prediction. Building upon the experiments in the previous section, we integrate attention method with models using deep contextual integration vectors as inputs, to analyze the influence of attention models on emotion prediction. The results are presented in Table 8.

**Table 8:** Results of ablation experiments on attention model.

Methods	Precision(%)	Recall (%)	F1-socre (%)
ConvNet & CFVW & Attention	81.17	79.84	80.03
ConvNet & CFVF & Attention	81.6	79.97	80.52
Bi-LSTM & CFVW & Attention	81.54	81.67	81.8
**Bi-LSTM & CFVF & Attention**	**81.57**	**82.7**	**81.15**

Combining the data from Table 7, Table 8, it is evident that incorporating attention models can effectively enhance performance. Specifically, in terms of F1-score, ConvNet & CFVW & Attention improved by 1.6 % compared to ConvNet & CFVW; ConvNet & CFVF & Attention increased by 1.65 % compared to ConvNet & CFVF; Bi-LSTM & CFVW & Attention enhanced by 1.96 % compared to Bi-LSTM & CFVW; and Bi-LSTM & CFVF & Attention showed an improvement of 1.8 % compared to Bi-LSTM & CFVF. This improvement is attributed to the attention models' ability to allocate more focus to highly relevant content in social media texts, thereby extracting more significant semantic features.

#### 4.5.3 Impact of deep parallel strategy

This section validates the effectiveness of the proposed DPCAF model in emotion prediction. Building upon our previous experiments, we compare the dual-channel models constructed by concatenating ConvNet & CFVW & Attention with Bi-LSTM & CFVW & Attention, and ConvNet & CFVF & Attention with Bi-LSTM & CFVF & Attention, against the final DPCAF model. This comparison aims to analyze the effectiveness of the deep parallel strategy, i.e., the multi-channel operation. The results are shown in Table 9.

From Table 9, it is clear that DPCAF achieves the best experimental results. Specifically, in terms of F1-score, DPCAF shows an improvement of 2.74 % over ConvNet & Bi-LSTM & CFVW & Attention, and 1.89 % over ConvNet & Bi-LSTM & CFVF & Attention. Additionally, combining the data from Table 8, it is observed that compared to single-channel models, DPCAF's F1-score significantly increases by 6.12, 5.63, 4.35, and 5 % over ConvNet & CFVW & Attention, ConvNet & CFVF & Attention, Bi-LSTM & CFVW & Attention, and Bi-LSTM & CFVF & Attention, respectively. This superior performance is attributed to DPCAF's ability to combine ConvNet and Bi-LSTM for extracting both local and global features, fully utilizing the contextual information in social media texts. Furthermore, the use of multi-feature fusion vectors as input enriches feature diversity. The deep parallel strategy based on multiple channels optimally leverages the semantic information in social media texts, thereby validating the effectiveness of the proposed DPCAF model in emotion prediction tasks.

#### 4.5.4 Impact of pooling strategy

To investigate the impact of different pooling strategies on model performance, this section selects average-pooling for ablation experiments, with results shown in Table 10.

As seen by comparing Table 9, Table 10, using the average-pooling strategy slightly decreases performance, but the reductions in Precision, Recall, and F1-score do not exceed 0.12 %. The reasons are as follows: although max-pooling can capture the most significant features, it may also miss some important information, especially when multiple lower intensity but related features jointly influence emotion judgment. Max-pooling tends to extract outputs from the most active neurons, ignoring smaller yet potentially important activations. This could lead to the neglect of subtle, dispersed emotional features, slightly impacting the model's comprehensiveness and precision.

**Table 9:** Results of ablation experiments on parallel strategy.

Methods	Precision(%)	Recall (%)	F1-socre (%)
ConvNet & Bi-LSTM & CFVW & Attention	82.95	82.5	83.41
ConvNet & Bi-LSTM & CFVF & Attention	83.07	82.49	84.26
**DPCAF**	**85.43**	**83.77**	**86.15**

**Table 10:** Results of ablation experiments on average-pooling strategy.

Methods	Precision(%)	Recall (%)	F1-socre (%)
ConvNet & Bi-LSTM & CFVW & Attention - average pooling	82.83	82.39	83.32
ConvNet & Bi-LSTM & CFVF & Attention -average pooling	82.88	82.3	84.18
**DPCAF-average pooling**	**85.39**	**83.67**	**86.09**

On the other hand, average pooling, by considering the average effect of all features, helps to capture these dispersed signals, potentially providing a more balanced perspective in some cases. Nevertheless, average-pooling might dilute key features, especially where there is significant feature variability. Therefore, while using max-pooling might miss some smaller signals, it generally better captures decisive, intense emotional features, which is beneficial for most emotion analysis tasks. In social media text analysis, even minor performance improvements can significantly impact practical applications, making max-pooling our preferred pooling strategy.

## 5 Conclusion

The proposed DPCAF method significantly enhances the emotional prediction performance in social media texts, particularly in the context of community wellness communications. The framework's innovative approach to integrating diverse word embeddings with part-of-speech and locational representations, combined with the use of deep parallel layers comprising ConvNet and Bi-LSTM, and the application of attention models, has demonstrated substantial improvements over both benchmark and state-of-the-art models. The results underscore the efficacy of DPCAF, evidenced by notable increases in Precision, Recall, and F1-score metrics. It should be noted, however, that social media posts often include images or videos alongside textual content, yet most current emotion prediction methods focus predominantly on text data, overlooking the emotional analysis of images and videos. Future research will aim to address this gap by integrating multi-modal short text dynamic semantical features from social media texts, images, and audio. Additionally, the adoption of capsule networks is planned to minimize the loss of emotion information. These enhancements are expected to more fully leverage the deep emotional features of social media short texts, thereby further improving the effectiveness of emotion analysis in social media contexts.

However, it's important to acknowledge certain limitations within our study. While DPCAF excels in analyzing textual content, it currently overlooks the emotional analysis of images and videos often present in social media posts. Future research endeavors should aim to address this gap by integrating multi-modal short text dynamic semantical features from social media texts, images, and audio. Additionally, the adoption of capsule networks is planned to mitigate the loss of emotion information, further enhancing the model's effectiveness.

Moving forward, our research will continue to explore avenues for improvement and expansion. Specifically, future studies will focus on refining the integration of multi-modal data sources and leveraging capsule networks to enhance emotion analysis in social media contexts. Additionally, efforts will be directed towards addressing potential scalability issues and optimizing the computational efficiency of the proposed framework. These advancements will contribute to a more comprehensive understanding of emotional dynamics in social media discourse and facilitate the development of more effective emotion prediction models.

## Data availability statement

Data will be made available on request.

## Ethics declarations

Review and/or approval by an ethics committee was not needed for this study because our research did not involve any ethical concerns.

## CRediT authorship contribution statement

**Feng Liu:** Writing – review & editing, Writing – original draft, Methodology. **Kun Hou:** Writing – review & editing, Methodology. **Yang Dong:** Writing – review & editing, Supervision.

## Declaration of competing interest

The authors declare that they have no known competing financial interests or personal relationships that could have appeared to influence the work reported in this paper.
